# Ultrasonic Image Feature Analysis under Deep Learning Algorithm to Evaluate the Efficacy of Drug-Coated Balloon for Treatment of Arteriosclerotic Occlusion

**DOI:** 10.1155/2022/3176716

**Published:** 2022-05-31

**Authors:** Yuchao Zhang, Gang Xu, Maozhen Chen, Ziliang Chen, Mingyang Shen, Ping Wang

**Affiliations:** Department of the Vascular Surgery, The Affiliated Huaian No.1 People's Hospital of Nanjing Medical University, Huaian City 223300, China

## Abstract

In order to explore the adoption of ultrasonic images under deep learning (DL) algorithm to evaluate the efficacy of drug-coated balloon (DCB) for treatment of arteriosclerotic occlusion, 56 patients who underwent DCB surgery of lower limb artery were selected and all the patients received the examinations of algorithmic ultrasound and digital subtraction angiography (DSA) before surgery. According to the examination methods, they were classified into algorithmic ultrasound group and DSA group. One to two months after DCB surgery, ultrasound examination was performed with the region-based faster convolutional neural network (faster R-CNN) target detection algorithm to check the therapeutic effect. The results showed that the image effect processed by the target detection algorithm based on DL was signally better than that of traditional ultrasonic processing algorithm in Dice, precision (Pre), and sensitivity, with significant difference (*P* < 0.05). Compared with DSA, algorithmic ultrasound showed better consistency between the two groups in the diagnosis of common femoral artery, superficial femoral artery, and popliteal artery stenosis, with statistical significance (*P* < 0.05). However, for the diagnosis of anterior tibial artery stenosis, the consistency between algorithmic ultrasound and DSA was general. The residual stenosis of each artery segment decreased obviously in postoperative review compared with that before surgery, and the difference was statistically significant (*P* < 0.05). Besides, both the pulsatility index (PI) and the blood flow velocity of the dorsalis pedis artery increased after surgery, compared with those before surgery, with significant differences (*P* < 0.05). To sum up, ultrasound based on DL target detection algorithm had good imaging effect and good consistency with DSA, which was of the clinical reference value. Additionally, DCB surgery was helpful to treat arteriosclerosis occlusion and improve limb blood supply, which had clinical adoption value.

## 1. Introduction

Lower extremity arteriosclerosis obliterans (LEASO) is a manifestation of systemic atherosclerosis in lower extremity arteries [1]. LEASO has a serious impact on people's normal life. With the aging of the global population and the improvement of the quality of people's daily life, the incidence of LEASO is increasing year by year. At present, the preoperative examinations of LEASO included lower limb angiography, digital subtraction angiography (DSA), and computed tomography angiography (CTA). All these methods can determine the location and severity of lower limb artery lesions, but each of them has its inherent limitation [2]. Arterial ultrasonography of lower limbs is simple and rapid, which is the first choice for clinical examination at present. The development effect of CTA imaging on distal arterioles is not very good [3]. DSA is currently the gold standard for diagnosing LEASO, but it requires the use of contrast agents. However, the risk of contrast agent-related complication is 10%, and the risk of death is 0.16%. Compared with other methods, ultrasound is the most simple, convenient, and inexpensive. Nevertheless, traditional ultrasound also has such limitations as the poor display effect of deep and small blood vessels due to slow blood velocity, which cannot precisely reflect the situation of blood vessels [4].

In recent years, with the rapid development of artificial intelligence (AI) technology, the combination of AI and medical imaging produces the intelligent diagnosis, that is, AI plays a central role and the deep training on the computer is for evaluation. Deep learning (DL) is a vital foundation that supports the progress of AI algorithm. DL is “deep” because it has many layers of nonlinear operations. Through deep network structure, DL can present accurate features, describe complex data, and greatly enhance the ability of fitting complex models. DL solves the problem of limited modeling and representation capabilities of traditional machine learning (ML).

Currently, the commonly used treatment methods for ASO include drug therapy, traditional surgical bypass, endovascular intervention, and stem cell transplantation. Percutaneous transluminal angioplasty (PTA) is one of the most common and representative techniques [5, 6]. However, massive clinical studies suggested that the restenosis rate of ASO treated by PTA is as high as 50%, so currently, PTA alone is rarely used in clinical treatment of ASO [7, 8]. Bare metal stent (BMS) arises as a remedy for PTA. It can improve the clinical efficacy of PTA when applied to residual stenosis, elastic retracement of tube wall, or flow-limiting interlayer. However, with the extensive application of stents, vascular intima is stimulated and elastic hyperplasia of intima is induced, which further leads to the occurrence of restenosis in stents. If stent fracture occurs, the patient will also have symptoms like lower limb bleeding again [9, 10]. Therefore, how to reduce the implantation of bare metal stents while improving long-term clinical efficacy has always been the focus of clinical research. The emergence of drug-coated balloon (DCB) provides a new direction for the treatment of lower extremity sclerosis occlusion. DCB can apply antiproliferative drugs to the surface of balloon catheter, thereby inhibiting intima hyperplasia and reducing restenosis. Abundant clinical studies showed that DCB has shown satisfactory results in the new stenosis or stent restenosis of coronary heart disease. However, its application in the treatment of lower extremity arteriosclerosis obliterans is still in its infancy. Foreign prospective studies pointed out that DCB technology is superior to PTA in one-year vessel patency rate and reintervention rate without target vessels. However, DCB technology in China is still in its infancy.

Modern medicine is highly dependent on imaging technology. The key to accurate diagnosis of disease lies in high-quality medical imaging and accurate impact diagnosis. In recent years, medical imaging equipment has been continuously improved and updated, and the imaging speed and quality have been significantly improved. However, the diagnosis of disease has always depended on experts to make it manually. The whole working process is time-consuming and labor-intensive, and it is easy to be misdiagnosed due to its subjectivity. In recent years, with the continuous development and progress of computer network technology, the auto-aided diagnosis method based on computer diagnosis technology has gradually become a research hotspot. Deep learning algorithm is widely used in this field [11]. In recent years, more attention has been paid to the faster R-CNN algorithm, which has achieved good results in a series of computer vision tasks such as image classification, target detection, and segmentation. Compared with traditional machine learning algorithms, faster R-CNN can directly input pixel data and optimize parameters in an end-to-end manner. Therefore, faster R-CNN can automatically learn feature expression directly from the provided samples, thus avoiding the complex image preprocessing and professional feature extraction process. Although the faster R-CNN algorithm has many advantages, it also has disadvantages. For example, with the deepening of layers, the difficulty of network training also increases. In addition, although faster R-CNN has good robustness, it lacks local information description, so it cannot solve the problem of local detail classification image. However, the differences between medical images tend to focus on local areas of focus. Therefore, how to use the faster R-CNN algorithm to solve this kind of problem still needs further in-depth research [12, 13].

To sum up, the adoption of ultrasound imaging based on the algorithms to evaluate the curative effect of DCB in the treatment of arteriosclerotic obliterans was investigated. Patients treated with arterial DCB of lower limbs were selected. The detection results of ultrasound based on the DL target detection algorithm, conventional ultrasound, and DSA were compared, and the algorithmic ultrasound was adopted to follow up the patients, aiming to provide a certain reference value for the clinical evaluation of the therapeutic effect of DCB and the selection of surgical treatment for arteriosclerotic occlusion.

## 2. Methods

### 2.1. Objects of Study

114 patients with lower limb artery DCB treatment in hospital from January 2018 to June 2020 were selected. After the patients who received the surgery not for the first time, were unwilling to participate, or did not review on time for other reasons were excluded, 56 patients were eventually included. There were 38 males and 18 females whose ages ranged from 51 to 79 years old, with an average age of 64.3 ± 7.64 years old. The conditions of lesion sites were as follows. There were 6 patients with common femoral artery, 36 patients with superficial femoral artery, 38 patients with popliteal artery, 30 anterior tibial artery, 6 patients with posterior tibial artery, and 4 patients with peroneal artery. All the patients received the examinations of algorithmic ultrasound and DSA before surgery. According to the examination methods, they were classified into algorithmic ultrasound group and DSA group. Another 3 patients were randomly selected for conventional ultrasound examination. Algorithmic ultrasound examination was performed at about 2 months after DCB surgery, and the therapeutic effect was checked. All the enrolled patients signed the informed consent and this study had been approved by the ethics committee of the hospital.

Inclusion criteria are as follows: patient age ≥ 18 years; patients diagnosed as peripheral vascular disease, intermittent claudication, or resting pain and other symptoms; imaging examination suggested superficial femoral artery or popliteal artery lesions; patients with first onset, no history of vascular surgical treatment or non-initial cases, who had undergone vascular surgery or endovascular treatment, and had recurrent luminal stenosis after surgery.

Exclusion criteria are as follows: patients allergic to contrast agents or unable to tolerate antiplatelet drugs; women who were pregnant or breast-feeding; intraoperative angiography indicated severe calcification; patients suffering from active bleeding or severe liver or kidney insufficiency cannot tolerate surgical treatment.

### 2.2. The Examination Methods

#### 2.2.1. The DSA Examination

Digital subtractive angiography X-ray machine was employed. Mark V Provis high-pressure syringe was also employed. The nonionic contrast agent and iohexol (300 mg/mL) were used. Routine allergy tests were implemented before surgery. The femoral artery was punctured with the Seldinger technique, and after successful intubation, the catheter sheath was inserted into the guide wire and angiography catheter. After systemic heparinization by injection of heparin according to patient's weight, intubation was performed to the proximal end of arterial occlusion by fluoroscopy. The patient was asked to hold the breath. The angiography of the associated arteries was performed with a high-pressure syringe injected with iohexol through a catheter (parameters : flow *F* = 5 mL/s, total amount of contrast agent TV = 15 mL, and pressure *P* = 300PSI).

#### 2.2.2. The Ultrasound Examination

Color Doppler ultrasound diagnostic instrument was employed. Lower limb artery probe frequency was 5 ~ 12 MHz, intra-abdominal iliac artery probe frequency was 2 ~ 4 MHz, sampling volume was 1 ~ 2 mm, and acoustic beam and included angle was below 60°. If the lower limb was swollen and the probe showed unclear lower limb arteries, the abdominal convex array probe (2-4 MHz) was used for supplementary examination. The color velocity scale was adjusted according to the actual blood flow image, and the wall filter was adjusted to remove the interference signal. A sampling ruler was placed in the center of the lumen parallel to the direction of blood flow, with a volume of 1-2 mm. If the artery was narrowed, it was placed in the narrowest place, and the angle between the acoustic beam and the direction of blood flow was less than or equal to 60°. Patient was placed in supine or prone position to check each artery. If patient was inconvenient to change the position, the external rotation booth was taken. When the dorsal foot artery was examined, the patient was asked to bend his lower limbs in supine position. After the common femoral artery was determined by transverse cutting from below the inguinal ligament, it was followed distally to the bifurcation of the common femoral artery. Then, the proximal and distal segments of the superficial femoral artery to the transitional part, the proximal segment of the deep femoral artery, the popliteal artery, and the calf artery were probed. When a certain segment of artery was examined, two-dimensional gray scale imaging and color flow imaging were used to locate the stenosis segment and predict the length of occlusive segment. The blood flow was assessed by short-interval multipoint sampling, and the degree of stenosis was graded based on the spectrum.

### 2.3. The Assessment of Results

#### 2.3.1. The Assessment of DSA

According to the physiological and anatomical sites, the lower limb arteries were classified into common femoral artery, superficial femoral artery, anterior tibial artery, and popliteal artery. The images were analyzed by experienced physicians to check the arterial wall, collateral circulation of the stenosis, and occlusion segment, and the stenosis and normal vessel diameter were measured. Stenosis rate = (normal inner diameter of proximal stenosis − diameter of proximal stenosis)/normal inner diameter of proximal stenosis × 100%.  Table 1 shows that each segment of blood vessel was scored. If there were more than one lesion in the same vessel, the highest stenosis rate was as the criterion. The superficial femoral artery with or without collateral circulation was statistically analyzed.

#### 2.3.2. The Assessment of Ultrasound

The artery intima-media thickening, the size, nature, and quantity of sclerosis plaque, arterial flow and blood flow, and the extent and degree of lesions were observed in the images. The specific parameters were collected, such as peak systolic velocity (PSV) at stenosis, before stenosis, and after stenosis. Support vector regression (SVR) was calculated (SVR = PSV stenosis/PSV proximal). The “proximal stenosis normal artery” of the arteries of the extremities referred to the same artery. The PSV of arteria dorsalis pedis and the pulsatility index (PI) were calculated. In Table 2, the stenosis rate referred to the stenosis degree of the obtained arteries, and the stenosis degree of each vessel segment was scored. If there were multiple lesions in the same vessel, the highest stenosis rate was as the standard. The superficial femoral artery with or without collateral circulation was statistically analyzed.

### 2.4. The Faster Region-Based Convolutional Neural Network (Faster R-CNN) Target Detection Algorithm

Faster R-CNN is a DL target detection algorithm based on candidate region extraction, feature extraction, and classification.  Figure 1 shows the detection principle. The input of the detection network is the image to be detected and a series of candidate target regions. The image to be detected is abstracted by deep convolutional neural network (Deep ConvNet) composed of multilayer convolution and maximum pooling to generate a convolutional feature map (Conv feature map). The auxiliary algorithm flowchart of the faster R-CNN algorithm in ultrasonic image processing is shown in Figure 2. The faster R-CNN algorithm model is shown in Figure 3.

The performance of each candidate target on the feature map is sent to the region of interest (ROI) pooling layer. The ROI pooling layer unifies these features as a fixed size feature to form a unified feature vector. If a feature of size *w*^∗^*h* is hoped to be obtained, for an input of arbitrary size *W*^∗^*H*, the ROI layer will classify the input into *W*/*w*^∗^*H*/*h* cells. Then, the maximum of all pixels in each cell is as the output of that cell. Fixed eigenvectors are sent to two independent output layers through the fully connected layer in turn. One is classifying the feature vectors corresponding to the target candidate region on each original image, and the other is performing accurate regression on the spatial position of the target candidate region on each original image.

In the classification layer, the multitask cost function Softmax is innovatively proposed to replace the traditional multidichotomy support vector machine (SVM) cascade to achieve the multiclassification. Softmax regression is namely the logistic regression under multiple categories. A data set {(*x*^(1)^, *y*^(1)^), (*x*^(2)^, *y*^(2)^), ⋯, (*x*^(*n*)^, *y*^(*n*)^)} is composed of *n* samples, where *x*^(1)^ ∈ *R*^(m + 1)^ is the sample feature, dimension is *m* + 1, and the class label is *y*^*i*^ ∈ {1, 2, ⋯, N}, namely, the *N* class. Equation (1) shows the hypothesis function of Softmax, and the model parameter is *θ*_1_, *θ*_1_, ⋯, *θ*_*k*_ ∈ *R*^(n + 1)^.

(1) $$\begin{array}{c} h_{\theta }\left(x^{\left(i\right)}\right)=\left[p\left(y^{\left(i\right)}=\left[\begin{array}{c} 1\\ 2\\ \begin{array}{c} \vdots \\ N \end{array} \end{array}\right]\;|\;x^{\left(i\right)};\theta \right)\right]=\left[\begin{array}{c} e^{\theta_{1}^{T}x^{\left(i\right)}}\\ e^{\theta_{2}^{T}x^{\left(i\right)}}\\ \begin{array}{c} \vdots \\ e^{\theta_{N}^{T}x^{\left(i\right)}} \end{array} \end{array}\right]/\overset{N}{\underset{j=1}{\sum }}e^{\theta_{j}^{T}x^{\left(i\right)}}. \end{array}$$

Equation (2) shows the cost function of Softmax regression and also shows the expansion of the cost function of dichotomy logistic regression. When 1{actual expression} = 1, it is 0 otherwise.

(2) $$\begin{array}{c} J\left(\theta \right)=-\frac{\left[\sum_{i=1}^{n}\sum_{j=1}^{N}1\left\{y^{\left(i\right)}=j\right\}\log\left(e^{\theta_{j}^{T}x^{\left(i\right)}}/\sum_{i}^{k}e^{\theta_{i}^{T}x^{\left(i\right)}}\right)\right]}{n}. \end{array}$$

At present, the gradient descent method is mostly used to minimize the cost function, and equation (3) shows the gradient equation derived from the cost function.

(3) $$\begin{array}{c} \nabla_{\theta_{j}}J\left(\theta \right)=-\frac{\sum_{i=1}^{n}\left[x^{\left(i\right)}\left(1\left\{y^{\left(i\right)}=j\right\}-p\left(y^{\left(i\right)}=j\;|\;x^{\left(i\right)};\theta \right)\right)\right]}{n}. \end{array}$$

During the training, parameters are optimized according to equation (4) every time.

(4) $$\begin{array}{c} \theta_{j}≔\theta_{j}-\alpha \nabla_{\theta_{j}}J\left(\theta \right)\left(j=1,\cdots ,N\right). \end{array}$$

The Softmax classification layer outputs the discrete probability distribution *R* = *r*_0_, ⋯, *r*_*N*_ of the target (each ROI) on the *S* + 1 category, and *r* is the calculated *S* + 1 output. The regression layer is strictly called the boundary box regression layer. Its function is adjusting and optimizing the position of candidate regions, and it follows R-CNN output *t*^*N*^ = (*t*_*x*_^*N*^, *t*_*y*_^*N*^, *t*_*w*_^*N*^, *t*_*h*_^*N*^) by definition. For *S* object categories, *N* is the object index. *t*^*N*^ represents the scale-invariant translation and logarithmic space height/width offset relative to the candidate region relative to the target real region.

Each training candidate region is marked with a true category *e* and an actual regression box *ν*. Equation (5) shows that multitask loss *L* is used for each candidate region to combine training classification and bounding box regression.

(5) $$\begin{array}{c} L\left(r,e,t^{u},v\right)=L_{\text{cls}}\left(r,e\right)+\lambda \left[e\geq 1\right]L_{\text{loc}}\left(t^{e},v\right). \end{array}$$

The loss function corresponding to the classification part is defined as equation (6).

(6) $$\begin{array}{c} L_{\text{cls}}\left(r,e\right)=-\log p_{e}. \end{array}$$

The *L*_*loc*_ is defined on the tuple of the actual bounding box regression target of class *e*, *v* = *v*_*x*_, *v*_*y*_, *v*_*w*_, *v*_*h*_. When *e* ≥ 1, the result is 1, and it is 0 otherwise. The background class is typically labeled *e* = 0. Equations (7) and (8) show the bounding box regression loss function.

(7) $$\begin{array}{c} L_{\text{loc}}\left(t^{e},v\right)=\underset{i\in \left\{x,y,w,h\right\}}{\sum }{\text{smooth}}_{L_{1}}\left(z_{i}^{e}-v_{i}\right), \end{array}$$

(8) $$\begin{array}{c} {\text{smooth}}_{L_{1}}\left(x\right)=0.5x^{2},\text{if}\left|x\right|<1;{\text{smooth}}_{L_{1}}\left(x\right)=\left|x\right|,\text{otherwise}. \end{array}$$

The hyperparameter *λ* function is used to control the balance between the two task losses. The idea of regional candidate extraction network is extracting candidate regions by sharing features extracted from convolutional neural network, thus saving the process of designing features separately during candidate region extraction. Multiple region candidate boxes are sent into the classification layer (cls layer) responsible for recognition and the regression layer (reg layer) responsible for the border of the regression candidate region. Through these definitions, the multitask loss function in Fast R-CNN is defined as shown in equation (9).

(9) $$\begin{array}{c} L\left(\left\{r_{i}\right\},\left\{z_{i}\right\}\right)=\frac{\sum_{i}L_{cls}\left(r_{i},r_{i}^{*}\right)}{N_{cls}}+\frac{\lambda }{N_{reg}}\underset{i}{\sum }p_{i}^{*}L_{reg}\left(z_{i},z_{i}^{*}\right). \end{array}$$

In equation (9), *i* is the index of the anchor point, *r*_*i*_ is the confidence degree of the anchor point as the foreground, and *r*_*i*_^∗^ is the actual classification of the anchor point. If the anchor point >0, the value is 1, and it is 0 otherwise. *z*_*i*_ is the vector composed of 4 coordinates after the prediction frame is parameterized. *z*_*i*_^∗^ is the actual bounding of the positive anchor point. The classification cost function *L*_*cls*_ is the logarithmic cost of the two categories, and equation (10) shows the regression cost function.

(10) $$\begin{array}{c} L_{reg}\left(z_{i},z_{i}^{*}\right)=R\left(z_{i}-z_{i}^{*}\right). \end{array}$$

In equation (10), *R* is defined as smooth_*L*_1__ in Fast R-CNN. These two terms are unified by *N*_reg_ and *N*_*cls*_ and weighted by the equilibrium parameter *λ*. The classification terms are unified by the minimum batch size (*N*_cls_ = 256), and the regression part is unified by the number of anchor points, which is about 2400.

### 2.5. The Index of Image Evaluation

The precision (Pre), Dice coefficient, and sensitivity [16] were used to evaluate. Equations (11), (12), and (13) show the calculations of these three indexes.

(11) $$\begin{array}{c} \text{Dice}=\frac{\left[2\left(\Omega Seg\cap \Omega Gr\right)\right]}{\left(\Omega Seg+\Omega Gr\right)}=\frac{2\text{TP}}{\left(2\text{TP}+\text{FP}+\text{FN}\right)}, \end{array}$$

(12) $$\begin{array}{c} \text{Precision}=\frac{\left(\Omega Seg\cap \Omega Gr\right)}{\Omega Seg}=\frac{\text{TP}}{\left(\text{TP}+\text{FP}\right)}, \end{array}$$

(13) $$\begin{array}{c} \text{Sensitivity}=\frac{\left(\Omega Seg\cap \Omega Gr\right)}{\Omega Gr}=\frac{\text{TP}}{\left(\text{TP}+\text{FN}\right)}. \end{array}$$

In equations (11), (12), and (13), *Qseg* represented the segmented tissue region, which was equal to TP + FP. *QGr* represented the standard tissue region, which was equal to TP + FN. TP represented the number of pixels that was correctly divided into positive classes in *Qseg*. TN represented the number of pixels that was correctly divided into negative classes in non-*Qseg*. *FP* represented the number of pixels that was incorrectly divided into positive classes in *Qseg*. *FN* represented the number of pixels that was incorrectly divided into negative classes in non-*Qseg*. The Dice coefficient represented the spatial coincidence degree between the tissue region and the standard tissue region. The Pre represented the proportion of pixels in a tissue region that was actually positive class. Sensitivity represented the proportion of what was correctly segmented in tissue regions. The evaluation values of the three indexes were all among 0-1. The larger the value was, the higher the consistency between *Qseg* and *QGr* was, and the better the segmentation effect was.

### 2.6. Statistical Method

SPSS 22.0 was employed for statistical analysis. Mean ± standard deviation ($\bar{x}$ ± *s*) was how measurement data were expressed. The two groups were compared by paired *t*-test. The consistency of the two examination methods was tested by *kappa*. The *χ*^2^ test was used to evaluate the collateral circulation of occlusive segment of artery. All the test levels were expressed as *a* = 0.05. The difference was statistically significant with *P* < 0.05.

## 3. Results

### 3.1. The Analysis of Ultrasonic Image Results

In Figure 4, the image effect processed by the target detection algorithm based on DL was signally better than that of traditional ultrasonic image processing algorithm in Dice, Pre, and sensitivity (*P* < 0.05).

### 3.2. Consistency Analysis of the Degree of Vascular Stenosis between the Two Examination Methods

When Kappa = 0.83 > 0.80 and *a* = 0.05, the consistency between the two groups was statistically significant (*P* < 0.05). The rate of common femoral artery stenosis in algorithmic ultrasound group had better consistency compared with that in DSA (Figure 5).

When 0.80 > Kappa = 0.74 > 0.60, *P* < 0.05, and *a* = 0.05, the consistency between the two groups was statistically significant. Compared with DSA, the rate of superficial femoral artery stenosis in algorithmic ultrasound group had better consistency (Figure 6).

When 0.80 > Kappa = 0.75 > 0.60, *P* < 0.05, and *a* = 0.05, the consistency between the two groups was statistically significant. Compared with DSA, the rate of popliteal artery stenosis in algorithmic ultrasound group had better consistency (Figure 7).

When 0.40 > Kappa = 0.37 > 0.20, *P* = 0.35 < 0.05, and *a* = 0.05, the consistency between the two groups was statistically significant. Compared with DSA, the consistency of the rate of anterior tibial artery stenosis in algorithmic ultrasound group was general (Figure 8).

### 3.3. Comparison of Shallow Branch Circulation between the Two Examination Methods

In the 56 cases of superficial femoral artery segmental occlusion and collateral circulation, there was no difference in collateral circulation between algorithmic ultrasound group and DSA group (Figure 9).

### 3.4. The Analysis of the Success Rate of Target Vascular DCB Surgery by Algorithmic Ultrasound

Compared with the conditions of the preoperative stenosis, the postoperative stenosis of superficial femoral artery was reduced to 4 cases, the postoperative residual stenosis was reduced to 2 cases, and the postoperative stenosis of anterior tibial artery was reduced to 6 cases (*P* < 0.05) (Figure 10).

Compared with the condition before surgery, PI of arteria dorsalis pedis increased after the surgery (*t* = −2.548, *P* < 0.05). The blood flow velocity of arteria dorsalis pedis also increased after the surgery (*t* = 12.721, *P* < 0.05) (Figure 11).

## 4. Discussion

LEASO is a local manifestation of systemic arteriosclerosis in the limb. Arteriosclerosis plaque, abnormal changes in the middle of the artery, and thrombosis can cause arterial lumen stenosis or even occlusion, thus causing intermittent claudication, gangrene, numbness, and chills [14, 17, 18]. Most of the patients are elderly, and the prevalence rate is higher in males than that in females. 38 male and 18 female patients were selected, whose ages ranged from 51 to 79 years old, with an average age of 64.3 ± 7.64 years old. DSA image is clear and accurate and image interference is small. Consequently, it is the gold standard for diagnosing the degree of arterial stenosis. However, it is an invasive examination, and the contrast agent has renal toxicity, so it cannot be repeated for many times. Hence, it cannot be used as a way of postoperative review [15, 16].

Ultrasound based on DL target detection algorithm was used to detect patients, which was compared with conventional ultrasound and DSA examination, and the accuracy of ultrasonic detection results of the algorithm was explored. The results showed that the image effect processed by the target detection algorithm based on DL was notably better than the traditional ultrasound image in Dice, Pre, and sensitivity (*P* < 0.05). The rate of common femoral artery stenosis in algorithmic ultrasound group was compared with that in DSA, and Kappa = 0.83. The rate of superficial femoral artery stenosis in algorithmic ultrasound group was compared with that in DSA, and Kappa = 0.74, which meant a good consistency. The rate of popliteal artery stenosis in algorithmic ultrasound group was compared with that in DSA, and Kappa = 0.75. The rate of anterior tibial artery stenosis in algorithmic ultrasound group was compared with DSA, and Kappa = 0.37 > 0.20, which meant that the consistency was general. There was no significant difference between algorithmic ultrasound group and DSA in evaluating collateral circulation in 56 patients with segmental occlusion of superficial femoral artery. Therefore, the detection results of the algorithmic ultrasound had certain reference value, but the difference of the DSA results was great sometimes, so it was not used only as the result of the diagnosis of arterial stenosis.

In the reexamination of the patients at 1-2 months after surgery, compared with the conditions before surgery, the postoperative stenosis of the superficial femoral artery was reduced to 4 cases, the postoperative residual stenosis of the artery was reduced to 2 cases, and the postoperative stenosis of the anterior tibial artery was reduced to 6 cases (*P* < 0.05). Compared with the condition before surgery, PI of the arteria dorsalis pedis increased after the surgery (*t* = −2.548, *P* < 0.05). The blood flow velocity of arteria dorsalis pedis also increased after the surgery (*t* = 12.721, *P* < 0.05). Hence, the blood supply to the distal end of the affected limb was improved, and DCB was helpful to effectively treat arteriosclerosis occlusion, which was of clinical adoption value. This was consistent with some previous research results [19, 20].

## 5. Conclusion

Compared with conventional ultrasound and DSA, ultrasound based on DL target detection algorithm had better imaging effect, and it had better consistency with DSA detection, which also had clinical reference value. Nevertheless, the accuracy needed to be improved, so it could not be used only as a diagnostic result of arterial stenosis. Moreover, DCB helped to treat arteriosclerosis occlusion effectively and improve limb blood supply, which had clinical adoption value. However, the number of cases included in this study is small, especially the segments of the peroneal artery and posterior tibial artery, which needs further investigation. Furthermore, the time and frequency of postoperative follow-up visit are few, which needs to be improved in the subsequent studies.

## Figures and Tables

**Figure 1:** The schematic diagram of Fast R-CNN detection.

**Figure 2:** Flow chart and example of auxiliary algorithm for ultrasonic image processing.

**Figure 3:** The Faster R-CNN model.

**Figure 4:** Comparison of ultrasonic image effect between the two groups. ^∗^Compared with traditional algorithm, *P* < 0.05.

**Figure 5:** Comparison of the degree of common femoral artery stenosis.

**Figure 6:** Comparison of the degree of superficial femoral artery stenosis.

**Figure 7:** Comparison of the degree of popliteal artery stenosis.

**Figure 8:** Comparison of the degree of anterior tibial artery stenosis.

**Figure 9:** Comparison of collateral circulation of superficial femoral artery.

**Figure 10:** The results of the success rate of DCB surgery. ^∗^Compared with that before operation, *P* < 0.05.

**Figure 11:** Comparison of PSV and PI of arteria dorsalis pedis before and after surgery. ^∗^Compared with the condition before surgery, *P* < 0.05.

**Table 1:** The diagnostic grading standards of DSA [14].

Degree of arterial stenosis	Arterial manifestation of DSA	Score
Normal	The wall of the tube was smooth and the lumen was not stenosis.	0
Degree I (mild)	The wall of the tube was normal or mildly irregular, and the lumen stenosis was 30%-49%.	1
Degree II (moderate)	Vascular stenosis was moderate, but there was no segmental absence of development, and the lumen stenosis was 50%-74%.	2
Degree III (severe)	Vascular stenosis was severe, with partial interruption of development, but the development occurred in the distal segment, with lumen stenosis ranging from 75% to 99%.	3
Degree V (occlusion)	There was no vascular development and occlusion was complete.	4

**Table 2:** The diagnostic grading standards of ultrasound [15].

Degree of arterial stenosis	PSV in the lesion (cm/s)	PSV ratio ^∗^	Score
Normal	<150	<1.5 : 1	0
30%-49% (mild)	150-200	1.5 : 1-2 : 1	1
50%-75% (moderate)	200-400	2 : 1-4 : 1	2
>75% (severe)	>400	>4 : 1	3
Occlusion	No blood flow signal	—	4

## Data Availability

The data used to support the findings of this study are available from the corresponding author upon request.
